The article "Children and Adolescent Dental Age Estimation by the Willems and Al Qahtani Methods in Surabaya, Indonesia" was published in 2022. Journal: Biomed Res Int.

# Children and Adolescent Dental Age Estimation by the Willems and Al Qahtani Methods in Surabaya, Indonesia

**DOI:** 10.1155/2022/9692214

**Published:** 2022-07-07

**Authors:** Beshlina Fitri Widayanti Roosyanto Prakoeswa, Arofi Kurniawan, An'nisaa Chusida, Maria Istiqomah Marini, Beta Novia Rizky, Mieke Sylvia Margaretha, Haryono Utomo, Anugerah I'zaaz Darmawan, Andini Kamilia Nur Aisyah, Aspalillah Alias, Otty Ratna Wahjuni, Anand Marya

**Affiliations:** ^1^Department of Forensic Odontology, Faculty of Dental Medicine Universitas Airlangga, Surabaya, Indonesia; ^2^Department of Basic Sciences and Oral Biology, Faculty of Dentistry, Universiti Sains Islam, Malaysia; ^3^Department of Dental Radiology, Faculty of Dental Medicine Universitas Airlangga, Surabaya, Indonesia; ^4^Department of Orthodontics, Faculty of Dentistry, University of Puthisastra, Phnom Penh, Cambodia; ^5^Center of Transdisciplinary Research, Saveetha Dental College, Saveetha Institute of Medical and Technical Science, Saveetha University, Chennai, India

## Abstract

**Objectives:**

Dental age estimation has been employed in a range of legal operations as well as catastrophe victim identification. Dental age estimation is regarded as an appropriate method for estimating a person's age because there is a high association between age and teeth. This study aims to assess the suitability of the Al Qahtani and Willems dental age estimation approaches for the Indonesian children and adolescent population.

**Methods:**

A total of 150 panoramic radiographs of patients (75 boys and 75 girls, 6-17 years old) were obtained from the Department of Radiology, Airlangga University, Indonesia. One researcher analyzed estimated dental age (EDA) twice in a one-week time-lapse using the Willems and Al Qahtani methods. The statistical analysis of the present study was carried out using IBM® SPSS® Statistics version 25.0 (IBM, Armonk, NY, USA).

**Results:**

The mean of this study's chronological age (CA) was 11.60 ± 3.41. Using the Willems method, the mean difference between CA and EDA for boys and girls was -0.41 ± 0.90. The mean difference between CA and EDA for boys and girls is 0.33 ± 0.61 using the Al Qahtani method.

**Conclusions:**

According to the findings of this investigation, the dental age estimation method proposed by Al Qahtani and Willems can be applied to the population in Surabaya. However, a comprehensive study is required when using this method because the data revealed significant statistical disparities between the two methods.

## 1. Introduction

Indonesia is the Pacific Ring of Fire's largest archipelagic country with hundreds of active volcanoes, causing a high vulnerability to natural disasters. Furthermore, natural and artificial disasters are affected by other elements such as climate change, geology, cultural diversity, and politics. Generally, disasters have had a profound impact on population numbers, health, and lifestyle. The disaster also causes severe injuries, deaths, food shortages, health facilities damage, and population movements [1, 2].

For many years, Indonesia has made global headlines due to devastating disasters that resulted in the deaths of many people and had a destructive effect on many aspects of life. In such situations, the Disaster Victim Identification (DVI) is a method for identifying mass catastrophe victims that must be applied to reveal the individual identity [3]. The primary importance of the identification process is finding the true identity of the victims. Positive identification is essential in human rights and correlated with religious and cultural aspects [4]. There are four significant aspects of biological identity in human identification: sex, age, stature, and ethnicity. In forensic and archeological contexts, age estimation is a critical parametric. Estimating age at death is critical for reconstructing a biological profile and thus enhancing the possibilities of identifying the human remains [5]. Lewis and Senn explained that authorities had used age estimation to narrow the search possibilities for unknown victims, estimate the age at death, distinguish cluster victims, determine eligibility for social benefits, and assist immigration agencies in processing undocumented immigrants [6–8].

Previous studies on dental age estimation found that the Willems and Al Qahtani methods showed high accuracy in heterogeneous populations. A reliable system for identifying victims in the case of a mass tragedy in Indonesia is urgently needed for millions of people from many cultures and religions [ 7, 9]. The current study sought to assess the applicability of the Willems and Al Qahtani methods in the Indonesian children and adolescent population.

## 2. Methods

The Institutional Ethical Committee has approved this study for the Health Research Faculty of Dental Medicine Universitas Airlangga (No.001/UN3.9.3/Etik/PT/2021). This cross-sectional study utilized panoramic radiographs from the Department of Radiology Dental Hospital Universitas Airlangga, Surabaya, 2016–2019. The study utilized 150 panoramic radiographs (75 males and 75 females, aged 6–17 years), which met the following inclusion criteria as follows:

- The available birthdate and radiographic recording date
- Good quality digital panoramic radiographs
- Clear radiographic image

The exclusion criteria are as follows:

- Panoramic radiographs with any pathological condition and/or tooth extractions
- Orthodontic appliances
- Congenital or developmental anomalies

The chronological age (CA), sex, and date of radiographic examination were tabulated in Microsoft®Excel®2019. These data were closed while determining the dental age to ensure a blinded study.

The panoramic radiographs were digitized and saved in JPEG format using a digital scanner. Microdicom DICOM viewer was used to process the digital panoramic radiographs. The estimated dental age (EDA) was calculated using the Willems and Al Qahtani methods. The Demirjian classification was used to evaluate the tooth development stage of all seven left mandibular teeth. Willems then converted each tooth's stage to a score and added them together to determine the EDA of the subject. The EDA was also examined using The London Atlas of tooth development proposed by Al Qahtani [10–12]. The measurement of dental age estimation was re-examined twice by the same observer at a one-week interval.

## 3. Results

The subjects of this study were divided into two groups based on sex and a certain age. The current study's statistical analysis was carried out utilizing IBM® SPSS® Statistics version 25.0 (IBM, Armonk, NY, USA). The inter-examiner reliability of the measurement was analyzed using the Cronbach Alpha coefficient. The significant differences between the chronological and estimated ages were calculated using paired *t*-test (*p*-value). The statistical significance was set at *p* < 0.05.

### 3.1. Overall Reliability Levels

A total of 150 panoramic radiographs (75 males and 75 females aged 6–17 years) were involved in this study. The average CA of males was 11.41±3.43 years, whereas female subjects were 11.79±3.39 years (Table 1). The Cronbach Alpha test was conducted to examine the inter-examiner agreement of tooth development stages scoring, with a coefficient of 0.6. The Kolmogorov-Smirnov test result showed the data was normally distributed and sufficient for additional statistical analysis, *p* > 0.05. The paired *t*-test was conducted to assess the differences between CA and EDA.

The paired *t*-test of Willems' method showed a significant difference between CA and EDA, with *p* < 0.05. Also, the overall mean difference in CA and EDA for males and females resulted in an underestimation of −0.40 ± 0.93 and−0.43 ± 0.88 years, respectively (Table 1). This finding suggested that a significant underestimation of age was observed in the Willems method.

The overall mean difference between CA and EDA while using the London Atlas of tooth development was 0.23 ± 0.53 for males and 0.42 ± 0.67 for females (Table 2). The paired *t-*test resulted in a significant overestimation in both sexes, with *p* < 0.05.

## 4. Discussion

Aging is related to the human body's growth and development process since it changes gradually with an organism's physical state. A person's age can be determined using a variety of characteristics, including bones and teeth. Teeth reveal a wide range of age estimation, from intrauterine to adult. However, the skeletal parameters show limitations, particularly for the middle-aged and adult population, because the growth process has ended [7, 13]. Estimating the age of death is critical in identifying the unknown deceased. Estimating a living person's age is also crucial in law enforcement proceedings [14].

Dental age estimation can be assessed morphologically, radiographically, histologically, and biochemically [15]. Radiographic examination for dental age estimation is an effective and low-cost method. Also, dental radiographic for dental treatment as antemortem data are readily available from the dental office. Panoramic radiographs were chosen for this study because they are thought to be the best approach for radiographic examination in children and adolescents, whereas intraoral x-rays are more challenging to apply in children [16]. Dental age estimation is considered the most accurate method because it shows a high correlation between age and teeth [15].

Various studies have examined the tooth development staging for dental age estimation. Willems suggested a novel approach to dental age estimation for the Belgian children population adapted from Demirjian's evaluation system. Willems' method showed improved accuracy in estimating chronological ages [9]. A study by Ismail et al., 2018, in the Malay population discovered that the Willems approach overestimated in ages 5 and 15. A study of the Willems method in Saudi children aged 4–16 years demonstrated a statistically significant distinction between EDA and CA [13]. The present study found that the Willems method significantly underestimated males and females in Indonesia [9]. This result was contrary to a study by Kurniawan et al., which claimed that there was no statistically significant difference between EDA and CA in males, whereas a similar result was found in the female population in Surabaya [14].

Al Qahtani et al. proposed the London tooth development atlas, which gives a wide range of dental age estimations. The subject of the Al Qahtani study was taken from two populations, European and Bangladeshi. The new atlas covered as much of the developing dentition as possible, and all ages were represented. The London Atlas accuracy has been evaluated in various demographics to guarantee that it is a global, practical, and all-encompassing method [10]. McCloe et al. used the London Atlas for age estimation in Hispanic children aged 6-15.99 years old. For the entire sample, the London Atlas showed a statistically significant value of overestimation in the population of Hispanic children, with a difference of +0.35 years (SD =0.89 years). The result of the present study corresponds with McCloe et al., and Ashraf et al.'s findings reveal a significant overestimation in age, with a difference of +0.33 years (SD =0.61 years) [13, 17]. This suggests that the growth and development of the dataset used in establishing Al Qahtani's technique differs from existing Surabaya population studies and that more research is needed to determine which element has a more significant impact on resulting in disparities in dental age [18].

The discrepancies in age estimation indicate a shift in children's overall development and suggest that nutrition may play a role in changes in dentition development [15]. Both inherent and external influences influence individual growth and development. Differences can strongly influence individuals' growth in food choices [18]. Fewer studies have been conducted to determine whether the timing of tooth development varies significantly across human populations. The persistent pattern of exaggerated ages observed by the published studies here implies that hereditary and environmental variables may impact variance in the timing of dental development [19, 20].

## 5. Conclusions

Results of this study imply that the dental age estimation approach proposed by Al Qahtani and Willems might be used for the Surabaya population. However, a detailed analysis is required when using this method because the results showed significant statistical differences in both methods. This could be due to the small number of subjects and age range that have been thought as few limitations as a result of this study. Further investigations with larger sample sizes will increase the dependability of the Willems and Al Qahtani approaches in Indonesia.

## Figures and Tables

**Table 1:** Descriptive analysis of CA, EDA, and age difference using the Willems dental age estimation method (age in years).

Gender	*N*	CA		EDA		Age difference			
		Mean	SD	Mean	SD	Mean	SD	Sig.	Remarks
Males	75	11.41	3.43	11.00	3.35	-0.40	0.93	0.000∗	Underestimated
Females	75	11.79	3.39	11.36	3.34	-0.43	0.88	0.000∗	Underestimated
Total	150	11.60	3.41	11.18	3.34	-0.41	0.90		Underestimated

∗Denotes a significant value.

**Table 2:** Descriptive analysis of CA, EDA, and age difference using the London Atlas of tooth development method (age in years).

Gender	N	CA		EDA		Age difference			
		Mean	SD	Mean	SD	Mean	SD	Sig.	Remarks
Males	75	11.41	3.43	11.64	3.40	0.23	0.53	0.000∗	Overestimated
Females	75	11.79	3.39	12.21	3.25	0.42	0.67	0.000∗	Overestimated
Total	150	11.60	3.41	11.93	3.33	0.33	0.61		Overestimated

∗Denotes a significant value.

## Data Availability

All data related to the study can be provided on reasonable request.

## Abbreviations

CA: Chronological age
EDA: Estimated dental age
IBM: International Business Machines
SPSS: Statistical Product and Service Solutions
JPEG: Joint Photographic Experts Group.
